# Long Noncoding RNA DSCAM-AS1 Facilitates Proliferation and Migration of Hemangioma Endothelial Cells by Targeting miR-411-5p/TPD52 Axis

This article has been retracted.

**DOI:** 10.1155/2022/8696432

**Published:** 2022-10-11

**Authors:** Yulong Wang, Shuiting Zhai, Jianwu Xing, Jinchi Zhang, Yingkun He, Guoquan Wang, Tianxiao Li

**Affiliations:** ^1^The Second Affiliated Hospital of Henan University of Science and Technology, Luoyang, 471000 Henan, China; ^2^Department of Vascular Surgery, The People's Hospital of Henan Province, Zhengzhou City, 450000 Henan Province, China; ^3^The First Affiliated Hospital of Fujian Medical University, Fuzhou, 350000 Fujian, China; ^4^Zhengzhou University People's Hospital, Henan Provincial People's Hospital and Henan Provincial Neurointerventional Engineering Research Center, Zhengzhou City, 450000 Henan Province, China

## Abstract

**Background:**

Diagnosed as a kind of vascular neoplasm of infancy, hemangioma (HA) occurs mainly due to the aberrant proliferation of endothelial cells. Existing evidence has manifested the close relationship of long noncoding RNAs (lncRNAs) with the pathogenesis of HA. Although lncRNA DSCAM antisense RNA 1 (DSCAM-AS1) has been revealed to be implicated in the progression of human diseases, the underlying mechanism DSCAM-AS1 exerts in HA formation is unclear.

**Aims:**

To figure out how DSCAM-AS1 may regulate the progression of human hemangioma endothelial cells (HemECs).

**Methods:**

DSCAM-AS1 expression was verified through RT-qPCR detection. Functional assays including EdU assay, colony formation assay, flow cytometry analysis, TUNEL assay, and transwell assay were applied to evaluate cell proliferation, apoptosis, and migration upon DSCAM-AS1 knockdown. Moreover, RNA pull-down assay, luciferase reporter assay, RIP assay, and other mechanism experiments were utilized for evaluating the correlation of DSCAM-AS1 and RNAs in HemECs.

**Results:**

DSCAM-AS1 knockdown inhibited proliferative capability and migratory capability of HemECs whereas expedited apoptosis. Molecular mechanism results testified DSCAM-AS1 could function as a ceRNA to bind miR-411-5p in HemECs. Besides, it was confirmed that tumor protein D52 (TPD52) served as a downstream target of miR-411-5p in HemECs. More importantly, related rescue assays uncovered that elevated expression of TPD52 or inhibited expression of miR-411-5p reversed the repressive progression of HemECs mediated by DSCAM-AS1 depletion.

**Conclusion:**

DSCAM-AS1 expedited HA progression via miR-411-5p/TPD52 pathway, which provided a novel therapeutic option for HA treatment.

## 1. Introduction

Hemangioma (HA) is a benign tumor commonly diagnosed in childhood, specifically in infants with low birth weight as well as premature infants. The etiology and pathogenesis of HAs have been investigated in recent years, but not completely clarified because of its complexity [1, 2]. Females are the majority of HA patients, with a female: male rate of approximately 3 : 1, and HA generally occurs about 14 days after birth [3, 4]. Severe HA results in a serous burden to patients and their beloved ones both physically and mentally, particularly on account of the disfigurement of skin lesions that severely influence the function of skin [3, 5]. Unfortunately, it is of great difficulty in treating severe HA, even with today's advances made in medical domain. Multiple researchers have been dedicated to studying and developing therapeutic strategies for HA, and advocate early diagnosis along with combined treatments so as to efficaciously limit HA growth and cut down the incidence of its complications [6]. What is more, it has been uncovered that the aberrant proliferation of endothelial cells is implicated in HA progression [7, 8]. Nevertheless, there is not much discussion on the molecular mechanism contributing to HA formation.

Long noncoding RNAs (lncRNAs) are identified as a group of transcripts with limited or no capacity of protein coding. Besides, lncRNAs are noncoding RNAs (ncRNAs) that possess longer than 200 nucleotides [9]. A previous study indicated that lncRNAs participate in a variety of biological courses, involving transcriptional and posttranscriptional regulation of genes, as well as epigenetics [10]. Abundant evidence has emphasized the importance of lncRNAs involvement in the occurrence and progression of diverse human tumors and diseases [11, 12]. More importantly, the critical regulatory effect of abnormally expressed lncRNA together with its molecular mechanism on the progression of HA has been manifested in many HA-related literatures. Among these molecular mechanisms, competing endogenous RNA (ceRNA) is the most documented. For example, lncRNA NEAT1 as a ceRNA promotes HA development via miR-361-5p/VEGFA axis [13]. LncRNA SNHG16 contributes to the proliferation, migration, and invasion of hemangioma endothelial cells (HemECs) via regulation of miR-520d-3p/STAT3 axis [14]. Recently, DSCAM antisense RNA 1 (DSCAM-AS1) has been recognized as an oncogenic lncRNA in breast cancer and elicits promoting effect on tumor growth [15]. It also contributes to the tumorigenesis of cervical cancer [16] and predicts a poor prognosis in ovarian cancer [17]. However, how DSCAM-AS1 may exert its functions in HA remains unknown, which arouses our interest.

In summary, our purpose is to clarify how DSCAM-AS1 may mediate HA development, and through relevant functional and mechanism experiments, we are going to verify the expression pattern of DSCAM-AS1 in HemECs and further uncover its potential function in the modulation of cell behaviors in HA progression. A series of rescue assays were taken to verify the interaction among involved RNAs in HemECs. We hope that what we have revealed through our research may shed some new lights on the researches of HA treatment.

## 2. Materials and Methods

### 2.1. Cell Samples

HemECs cell lines were commercially acquired from the Institute of Biochemistry and Cell Biology (Shanghai, China) and maintained under 5% CO_2_ and 37°C. Samples were cultured in Endothelial Basal Medium-2 (EBM-2) with 10% FBS and 1% Pen/Strep solution as supplements.

### 2.2. Total RNA Extraction and RT-qPCR

Total RNA extracted from human HA tissue and HemEC cell samples were achieved by TRIzol reagent (Invitrogen) as instructed by supplier. 1 mg of total RNA was used for cDNA synthesis applying PrimeScript™ RT Master Mix (TaKaRa, Shiga, Japan), and then SYBR® Premix Ex Taq^TM^ II kit (TakaRa) was applied for qPCR on the 7500 Fast Real-Time PCR System (Applied Biosystems, Foster City, CA). Relative target gene expression was calculated by 2^−∆∆Ct^ method with standardization to GAPDH or U6.

### 2.3. Plasmid Transfection

Specific shRNAs and the corresponding negative control (NC) were commercially acquired from Genepharma (Shanghai, China), which were applied for the depletion of DSCAM-AS1 and TPD52 in HemECs. The pcDNA3.1/TPD52 and pcDNA3.1, as well as the miR-411-5p mimics/inhibitor and NC mimics/inhibitor were all designed by RiboBio Co., Ltd. (Guangzhou, China). Transfection was performed for 48 h using Lipofectamine2000 (Invitrogen).

### 2.4. EdU Incorporation Assay

Proliferation of HemECs was detected using EdU incorporation assay with Click-iT® EdU Imaging Kits (Invitrogen) as guided by supplier. Cultured cell samples in 24-well plates were labeled with EdU for 2 h, then fixed and permeabilized. DAPI was added for 30 min for observing with fluorescence microscopy (Olympus, Tokyo, Japan).

### 2.5. Colony Formation

500 clonogenic cell lines in the 6-well plates were processed with the 14 days of incubation, then fixed and stained with 0.5% crystal violet. Clones were counted manually.

### 2.6. Flow Cytometer of Apoptosis

Cells in 6-well plates were trypsinized for resuspending in the Binding buffer adding the FITC-conjugated Annexin V and PI dye for 15 min at room temperature. Flow cytometer was employed with FACS Calibur (BD Bioscience, San Jose, CA).

### 2.7. Caspase-3 Measurement

The caspase-3 activity kit was procured from Beyotime (Shanghai, China) for the determination of caspase-3 activity in cell lysates as per the user manual. The microplate reader (Tecan, Männedorf, Switzerland) was used.

### 2.8. TUNEL Staining

TUNEL staining assay was conducted as per the instruction of One-Step TUNEL Apoptosis Assay Kit (Beyotime) for detecting the cell apoptosis. TUNEL-positive cells were determined by fluorescence microscopy.

### 2.9. Transwell Migration Assay

The 24-well transwell chambers were procured from Corning Incorporated (Corning, NY) for cell migration. 5 × 103 cells in serum-free medium were added into the upper chamber; the complete medium was added into the lower chamber. After 24 hours, cells in the bottom were all stained with crystal violet in 4% paraformaldehyde for observing.

### 2.10. Subcellular Fractionation

The lysed cell samples in cell fractionation buffer were collected to centrifuge for nucleus-cytoplasm separation. After removing supernatant, samples were processed with cell disruption buffer. DSCAM-AS1 expression level in nuclear and cytoplasmic fractions went through RT-qPCR analysis.

### 2.11. RNA Pull-down

RNA pull-down analysis was achieved using Pierce™ Magnetic RNA-Protein Pull-Down Kit (Thermo Fisher Scientific, Waltham, MA) in light of the guidebook. Protein extracts were mixed with DSCAM-AS1 biotin probe and magnetic beads. The pull-downs were analyzed by RT-qPCR.

### 2.12. Luciferase Reporter Assay

The constructed reporter plasmids pmirGLO-DSCAM-AS1-WT/Mut and pmirGLO-TPD52-WT/Mut were cotransfected into cultured HemEC cells for 48 h. Dual-Luciferase Reporter Assay System (Promega, Madison, WI) was employed for detection of fluorescence intensity changes as required by supplier.

### 2.13. RIP Assay

Using Magna RIP™ RNA Binding Protein Immunoprecipitation Kit (Millipore), RIP assay was conducted with the human anti-Ago2 and anti-IgG (Millipore). Precipitated RNAs were all estimated by RT-qPCR.

### 2.14. Statistical Analysis

Statistical analysis was achieved by SPSS 22.0 (IBM, Armonk, NY, USA) with significant level at *P* < 0.05, and data were all expressed as the mean ± SD. Prism version 5.0 (GraphPad Software, La Jolla, CA) was applied to generate images. Group comparison was performed with Student's *t* test and one-way ANOVA analysis. Bio-triple replications were required in each assay.

## 3. Results

### 3.1. Silenced DSCAM-AS1 Attenuates Cell Proliferation and Migration whereas Motivates Cell Apoptosis in HemECs

For purpose of researching the underlying function of DSCAM-AS1 on HA formation, we knocked down its expression in HemECs. After downregulating DSCAM-AS1 expression in HemECs utilizing sh-DSCAM-AS1#1/2 (Figure 1(a)), we performed a serious of functional assays. EdU assay illustrated that EdU positive cells were significantly decreased in the sh-DSCAM-AS1 transfection groups, suggesting cell proliferative capability was repressed by DSCAM-AS1 downregulation (Figure 1(b)). Further, it was illustrated from colony formation assay that cell colonies were reduced, which proved that cell proliferative capability could be repressed by DSCAM-AS1 knockdown (Figure 1(c)). Then flow cytometry analysis indicated that the cell apoptosis rate was significantly increased by the transfection of sh-DSCAM-AS1 (Figure 1(d)). Besides, caspase-3 activity was elevated in the transfection cell groups, which further confirmed the promotion of cell apoptosis ability (Figure 1(e)). It was further proved that the quantity of TUNEL positive cells was obviously increased by DSCAM-AS1 downregulation (Figure 1(f)). In the end, transwell assay was conducted to measure cell migration capability, and we discovered that after transfection, the number of migrated cells was decreased (Figure 1(g)). In short, silenced DSCAM-AS1 attenuates cell proliferation and migration whereas motivates cell apoptosis in HemECs.

### 3.2. MiR-411-5p is Targeted by DSCAM-AS1 in HemECs

Through subcellular fractionation analysis of DSCAM-AS1 distribution, we realized that DSCAM-AS1 was mainly scattered in the cytoplasm of HemECs, suggesting that DSCAM-AS1 may regulate gene expression via a posttranscriptional way (Figure 2(a)). Further, RIP assay proved that DSCAM-AS1 was bound to Ago2 protein (Figure 2(b)). As mostly documented, lncRNA mediates cancer progression by serving as microRNA (miRNA) sponge. Thus, we speculated that DSCAM-AS1 probably contributed to HA formation via binding to certain miRNA. Through starBase (http://starbase.sysu.edu.cn/) and DIANA (http://carolina.imis.athena-innovation.gr/diana_tools/web/index.php) database, 13 miRNAs were predicted to possess binding capacity with DSCAM-AS1 (Figure 2(c)). Subsequently, we observed that only miR-411-5p was conspicuously enriched in DSCAM-AS1 biotin probe group, confirming that miR-411-5p combined with DSCAM-AS1 in HemECs (Figure 2D). Besides, through starBase, a binding site between miR-411-5p and DSCAM-AS1 was predicted (Figure 2(e)). After elevated miR-411-5p expression in HemECs (Figure 2(f)), the luciferase activity of DSCAM-AS1-WT was markedly reduced whereas the luciferase activity of DSCAM-AS1-Mut presented no evident changes (Figure 2(g)). These results demonstrated that DSCAM-AS1 can sponge miR-411-5p via acting as a ceRNA.

### 3.3. MiR-411-5p Represses Cell Proliferation and Migration of HemECs

To study whether miR-411-5p elicit effect on HemEC progression, we employed gain-of-function assays. EdU staining assay and colony formation assay unveiled that miR-411-5p overexpression hampered cell proliferation (Figures 3(a) and 3(b)). Conversely, data from flow cytometry analysis, caspase-3, and TUNEL experiments verified the facilitating effect of miR-411-5p upregulation on cell apoptosis (Figures 3(c)–3(e)). Furthermore, transwell assay delineated that the migration ability of HemECs was suppressed by miR-411-5p overexpression (Figure 3(f)). Taken together, miR-411-5p represses cell proliferation and migration of HemECs.

### 3.4. TPD52 is a Downstream Target of miR-411-5p in HemECs

To further probe into the mechanism of DSCAM-AS1 in HemECs, we planned to find the target gene of miR-411-5p. After searching starBase under particular condition (CLIP − Data > = 5; pan − Cancer > = 10), some mRNA candidates were screened out (Figure 4(a)). In order to screen out the most suitable mRNAs, we performed luciferase reporter assay and found that only the luciferase activity of miR-411-5p–overexpressed HemECs was obviously declined in TPD52 group (Figure 4(b)). Further, after upregulating miR-411-5p expression or downregulating DSCAM-AS1 expression, TPD52 expression was remarkably decreased (Figures 4(c) and 4(d)). Thus, we selected TPD52 to conduct the further assays. To make further exploration of the interaction between miR-411-5p and TPD52, online search of starBase predicted the binding sites between them (Figure 4(e)). The luciferase activity of TPD52-WT, but not that of TPD52-Mut, was lowered after miR-411-5p expression was elevated in HemECs (Figure 4(f)). Subsequent analysis of RIP assay depicted that DSCAM-AS1, miR-411-5p, and TPD52 were enriched in anti-Ago2 group, testifying the coexistence of them in RISC (Figure 4(g)). Besides, TPD52 was significantly pulled down by the biotinylated miR-411-5p probe (Figure 4(h)). These results demonstrated that miR-411-5p could bind to TPD52.

To investigate the biological role of TPD52 in HemECs, we knocked down TPD52 prior for loss-of-function assays (Figure S1A). As displayed in Figure S1B-C, TPD52 downregulation impaired cell proliferation. Besides, cell apoptosis capability was enhanced by inhibiting TPD52 expression, as manifested by flow cytometry, TUNEL and caspase-3 expression detection (Figure S1D-F). What is more, the migration ability of HemECs was suppressed after TPD52 expression was reduced (Figure S1G). In brief, TPD52 is directly targeted by miR-411-5p in HemECs and it accelerates cell proliferation and migration.

### 3.5. DSCAM-AS1 Mediates HemEC Progression by Targeting miR-411-5p/TPD52 Axis

On the basis of the above results, we realized that DSCAM-AS1 could indirectly regulate TPD52 expression through binding to miR-411-5p. Herein, we wondered whether and how DSCAM-AS1/miR-411-5p/TPD52 pathway modulated the progression of HemECs. Prior to rescue assay to testify the probable mechanism of DSCAM-AS1, the overexpression efficiency of TPD52 and the inhibition efficiency of miR-411-5p were tested in HemECs, and the results appeared to be satisfactory (Figure 5(a)). Then, data obtained from EdU and colony formation assays suggested that miR-411-5p inhibition or TPD52 upregulation could countervail the suppressive effect of DSCAM-AS1 deficiency on the proliferation of HemECs (Figures 5(b) and 5(c)). Likewise, inhibiting miR-411-5p expression or elevating TPD52 expression could reverse the promoting function on cell apoptosis mediated by DSCAM-AS1 knockdown (Figures 5(d)–5(f)). Besides, the suppressed capacity of HemECs to migrate induced by DSCAM-AS1 downregulation could be recovered by miR-411-5p repression or TPD52 overexpression (Figure 5(g)). All in all, DSCAM-AS1 downregulation impairs HemEC progression via targeting miR-411-5p/TPD52 axis.

## 4. Discussion

Accumulating evidence has verified that lncRNAs exert significant function on different kinds of human diseases through ceRNA network, including HA. For instance, lncRNA H19 improves mesenchymal stem cells survival and their angiogenic capability though regulating miR-199a-5p/VEGFA axis [18]. LncRNA FTX targets miR-29b-1-5p and Bcl2l2 to modulate apoptosis of cardiomyocyte [19]. LncRNA CASC9 as a ceRNA mediates HA development via miR-125a-3p/Nrg1 pathway [20]. Although DSCAM-AS1 upregulation has been revealed to expedite breast cancer malignancy [15], the knowledge about whether and how DSCAM-AS1 regulate HA progression remains to be deciphered. In this study, we proved that DSCAM-AS1 downregulation could restrain the proliferation and migration of HemECs. These results confirmed that DSCAM-AS1 functioned as an oncogene in HA.

As largely uncovered, lncRNA as a ceRNA is involved in the progression of human malignancies and diseases via sponging miRNA and targeting mRNA [21–23]. According to the findings that DSCAM-AS1 located in cytoplasm of HemECs, we speculated that DSCAM-AS1 mediated HA formation though sponging miRNA. Through bioinformatics tools, we sifted out several miRNA candidates that may combine with DSCAM-AS1, but the RNA pull-down data later manifested that only miR-411-5p was conspicuously pulled down by DSCAM-AS1 biotin in HemECs. Furthermore, we proved that miR-411-5p alleviate the malignant cell behaviors in HemECs. MiR-411-5p, a miRNA previously investigated in multiple cancers, has been manifested to suppress non-small-cell lung cancer cell migration and invasion by inhibiting PUM1 expression [24] and inhibit breast cancer cell proliferation and metastasis via targeting GRB2 [25]. Previous studies have revealed DSCAM-AS1's involvement in cancer progression via ceRNA pattern. For example, DSCAM-AS1 aggravates non-small-cell lung cancer progression via sponging miR-577 to further modulate HMGB1 expression [26]. DSCAM-AS1 is regarded as a molecular sponge of miR-384 to modulate AKT3 expression, thereby aggravating colorectal cancer malignancy [27]. This is the first time that we have revealed the ceRNA interaction of DSCAM-AS1 and miR-411-5p on the progression of HA. Further, upregulation of miR-411-5p was verified to impair HA progression.

Tumor protein D52 (TPD52), an identified mRNA with protein coding potential, has been unveiled to function as an oncogene in human cancers. For example, TPD52 was highly expressed in colorectal cancer cells and correlated with poor prognosis [28]. TPD52 promoted cell growth in nasopharyngeal carcinoma [29]. Silencing of TPD52 inhibited the malignant cell behaviors in pancreatic cancer by deactivating Akt pathway [30]. Importantly, TPD52 was reported to take part in the cell growth and aggressiveness of HA [31]. In the current research, TPD52 expression in HemECs was validated to be negatively modulated by miR-411-5p but positively regulated by DSCAM-AS1. TPD52 was a direct target gene of miR-411-5p. Moreover, knockdown of TPD52 represses HemEC proliferation and migration. What is more, the inhibitive effect of DSCAM-AS1 downregulation on HemEC progression could be rescued by inhibiting miR-411-5p expression or elevating TPD52 expression.

## 5. Conclusion

DSCAM-AS1 elevates TPD52 expression to drive the progression of HA through sponging miR-411-5p. This finding provides evidence of DSCAM-AS1 promoting function on HA progression. Besides, the discovery of the DSCAM-AS1/miR-411-5p/TPD52 pathway suggests an innovative clue for HA treatment.

## Figures and Tables

**Figure 1:** Silenced DSCAM-AS1 attenuates cell proliferation and migration whereas motivates cell apoptosis in HemECs. (a) DSCAM-AS1 level in HemECs was tested by RT-qPCR. (b–c) The proliferation ability was measured by EdU and colony formation assays. (d–f) The apoptosis ability was measured by analyses of flow cytometry, caspase-3 activity, and TUNEL. (g) Cell migration capability was analyzed via transwell. ^∗∗^*P* < 0.01.

**Figure 2:** MiR-411-5p is targeted by DSCAM-AS1. (a) The subcellular distribution of DSCAM-AS1 was detected via subcellular fractionation assay. (b) RIP assay proved the combination of DSCAM-AS1 and Ago2 protein. (c) 13 miRNAs were predicted to possess binding capacity with DSCAM-AS1 via starBase and DIANA database. (d) The binding between DSCAM-AS1 and these miRNAs was tested by RNA pull-down. (e) A binding site between miR-411-5p and DSCAM-AS1 was predicted via starBase. (f) RT-qPCR was utilized to analyze the overexpression efficiency of miR-411-5p. (g) The binding of DSCAM-AS1 with miR-411-5p was validated via luciferase reporter assay.^∗∗^*P* < 0.01.

**Figure 3:** MiR-411-5p represses cell proliferation and migration of HemECs. (a–b) The proliferation ability was measured by EdU assay and colony formation assay. (c–e) The apoptosis ability of transfected cells was measured via flow cytometry analysis, caspase-3 activity assay, and TUNEL assay. (f) Cell migration capability was analyzed through transwell in cells transfected with miR-411-5p mimics or NC mimics.^∗∗^*P* < 0.01.

**Figure 4:** TPD52 is a downstream target of miR-411-5p in HemECs. (a) StarBase database predicted the possible mRNAs for miR-411-5p. (b) Luciferase reporter assay was applied for detecting the binding situation of miR-411-5p and possible mRNAs. (c–d) TPD52 level was analyzed in HemECs transfected with different plasmids. (e) A binding site between miR-411-5p and TPD52 was speculated though utilizing starBase. (f) The interaction between TPD52 with miR-411-5p was proven via luciferase reporter assay. (g) RIP assay confirmed the coexistence of DSCAM-AS1, miR-411-5p, and TPD52 in RISC. (h) RNA pull-down assay further proved the binding of miR-411-5p and TPD52. ^∗∗^*P* < 0.01.

**Figure 5:** DSCAM-AS1 mediates HemEC progression by targeting miR-411-5p/TPD52 axis. (a) The overexpression efficiency of TPD52 and the inhibition efficiency of miR-411-5p were tested in HemECs through RT-qPCR analysis. (b–c) The proliferation ability was determined by EdU and colony formation assays. (d–f) Cell apoptosis ability was measured through analyses of flow cytometry, caspase-3 activity, and TUNEL. (g) Cell migration capability in different groups was evaluated via transwell.^∗∗^*P* < 0.01.

## Data Availability

All data, models, and code generated or used during the study appear in the submitted article.

## Abbreviations

HA: Hemangioma
DSCAM-AS1: DSCAM antisense RNA 1
TPD52: Tumor protein D52
HemECs: Human hemangioma endothelial cells
lncRNAs: Long noncoding RNAs
ncRNAs: Noncoding RNAs
ceRNA: Competing endogenous RNA
miRNA: microRNA
FBS: Fetal bovine serum
RT-qPCR: Quantitative reverse transcription real-time polymerase chain reaction
EdU: 5-Ethynyl-2′-deoxyuridine
DAPI: 4′,6-diamidino-2-phenylindole
TUNEL: Terminal deoxynucleotidyl transferase (TdT) dUTP Nick-end labeling
RIP: RNA immunoprecipitation
WT: Wild-type
Mut: Mutant
SD: Standard deviation
ANOVA: Analysis of variance.

## Supplementary Materials

Supplementary Materials Figure S1: (a) the efficiency of TPD52 knockdown was evaluated via RT-qPCR. (b–c) The proliferation ability of HemECs transfected with sh-TPD52#1/2 or sh-NC was measured by EdU assay and colony formation assay. (d–f) The apoptosis ability was measured via flow cytometry analysis, caspase-3 activity assay, and TUNEL assay. (g) Cell migration capability was assessed through transwell in different groups.^∗∗^*P* < 0.01.
